# QbD-based rivastigmine tartrate-loaded solid lipid nanoparticles for enhanced intranasal delivery to the brain for Alzheimer's therapeutics

**DOI:** 10.3389/fnagi.2022.960246

**Published:** 2022-08-11

**Authors:** Deepshi Arora, Shailendra Bhatt, Manish Kumar, Ravinder Verma, Yugam Taneja, Nikita Kaushal, Abhishek Tiwari, Varsha Tiwari, Athanasios Alexiou, Sarah Albogami, Saqer S. Alotaibi, Vineet Mittal, Rajeev K. Singla, Deepak Kaushik, Gaber El-Saber Batiha

**Affiliations:** ^1^M.M. College of Pharmacy, Maharishi Markandeshwar (Deemed to be University), Ambala, Haryana, India; ^2^Guru Gobind Singh College of Pharmacy, Yamuna Nagar, Haryana, India; ^3^Department of Pharmacy, G.D. Goenka University, Gurugram, Haryana, India; ^4^Zeon Lifesciences Pvt. Ltd., Paonta Sahib, Himachal Pradesh, India; ^5^Pharmacy Academy, IFTM University, Moradabad, UP, India; ^6^Department of Science and Engineering, Novel Global Community Educational Foundation, Hebersham, NSW, Australia; ^7^AFNP Med Austria, Wien, Austria; ^8^College of Science, Taif University, Taif, Saudi Arabia; ^9^Department of Pharmaceutical Sciences, Maharshi Dayanand University, Rohtak, Haryana, India; ^10^Institutes for Systems Genetics, Frontiers Science Center for Disease-related Molecular Network, West China Hospital, Sichuan University, Chengdu, Sichuan, China; ^11^iGlobal Research and Publishing Foundation, New Delhi, India; ^12^Faculty of Veterinary Medicine, Department of Pharmacology and Therapeutics, Damanhour University, Damanhour, Egypt

**Keywords:** Alzheimer, intranasal, rivastigmine, CCD, pharmacokinetics, *ex vivo*, optimization

## Abstract

Alzheimer's disease (AD) is a neurodegenerative disease that affects a wide range of populations and is the primary cause of death in various countries. The treatment of AD is still restricted to oral conventional medicines that act only superficially. Fabrication of intranasal solid lipid nanoparticulate system for the uptake of therapeutic agents will act as a convincing approach with limited off-site toxicity and increased pharmacological activity. The objective of this study was to formulate, optimize, and evaluate the efficiency of rivastigmine tartrate (RT)-loaded intranasal solid lipid nanoparticles (SLNs) employing the solvent-evaporation diffusion method. To optimize the formulation parameters, the central composite design (CCD) was used. Lipid concentration (X1) and surfactant concentration (X2) were considered to be independent variables, while particle size (Y1), percentage entrapment efficiency (Y2), and percentage drug release (Y3) were considered as responses. The solid lipid was glyceryl monostearate, while the surfactant was polysorbate 80. The optimized formulation has a particle size of 110.2 nm, % entrapment efficiency of 82.56%, and % drug release of 94.86%. The incompatibility of drug excipients was established by differential scanning calorimetry (DSC) and Fourier-transform infrared spectroscopy (FTIR). Nasal histopathology tests on sheep mucosa revealed that the developed SLNs were safe to utilize for intranasal delivery with no toxicity. *Ex vivo* permeation investigations revealed that the flux and diffusion coefficients for RT solid lipid nanoparticles and RT solution were 3.378 g/cm^2^ /h and 0.310–3 cm^2^ /h, respectively. Stability studies demonstrated that the developed SLNs were stable when stored under various storage conditions. The viability and vitality of adopting a lipid particle delivery system for improved bioavailability *via* the intranasal route were also established in the *in vivo* pharmacokinetic investigations. According to the histopathological and pharmacokinetic investigations, the developed formulations were safe, non-lethal, efficient, and robust. These results suggest the potentiality provided by rivastigmine tartrate-loaded solid lipid nanoparticles for nasal delivery.

## Introduction

Alzheimer's disease (AD)/dementia is the most restrictive and progressively debilitating neurological condition affecting the aged population economically and socially. The key histopathological features of AD are the accumulation of extracellular amyloid plaques (AP) and neurofibrillary tangles in the brain. Studies have shown that soluble Aβ oligomers are more toxic to neurons than plaques (Iyaswamy et al., 2021). Recent findings hypothesize that abnormal phosphorylation of tau is a causative factor for sporadic AD before Aβ formation in the human brain. In AD, hyperphosphorylated tau proteins dissociate from microtubules and self-assemble into aggregates. It is an age-related disorder that is accompanied by a loss of memory and has manifestations like congestive heart failure. It is characterized by recent memory loss in the early stages accompanied by a profound cognitive decline in the later stages (Iyaswamy et al., 2022). Behavioral issues, loss of working abilities, impaired communication skills, poor reasoning power, and loss of personality traits are other hallmarks of this neurodegenerative disorder (Sreenivasmurthy et al., 2022).

In the case of central nervous system (CNS) disorder, traditional drug administration enters the brain through the systemic circulation. To achieve the appropriate therapeutic concentration at the target site, systemic drug levels must be increased through repeated dosage or prolonged administration. This could lead to an increase in toxicity. When systemic effects are desired, the oral route of medication delivery is regarded to be the most desirable and effective. Although the oral route has received a lot of attention for systemic drug administration, the limited oral bioavailability and first-pass metabolism of several active treatments have prompted researchers to look for a more efficient systemic delivery route. Recent advances have emphasized the opportunity of developing the nasal route of delivery for direct delivery of drug moieties from (N2B) nose to the brain in humans (Pardridge, 2005). In various studies performed on animal models and humans, it was observed that CNS delivery of drugs *via* the nasal route is largely dependent upon molecular weight and the lipophilicity of the drug (Illum, 2003). The intranasal route of drug administration overcomes the barrier existing between blood and brain (BBB) and provides direct entry into the brain without surgical intervention and ease of administration (Misra et al., 2003).

The only therapeutic class of drugs licensed for the symptomatic treatment of AD is cholinesterase (ChE) inhibitors. These medications improve cholinergic function by blocking acetylcholine (ACh) degrading enzymes, thus increasing the amount of ACh available to excite nicotinic and muscarinic receptors in the brain. Tacrine, donepezil, rivastigmine, and galantamine are the four ChE inhibitors currently approved for the symptomatic treatment of Alzheimer's disease. Although all of these drugs raise ACh levels in the brain, their pharmacological and pharmacokinetic profiles varied significantly; for example, enzymes inhibited potency, brain selectivity, chemical class, mode of action, metabolism, and dose-dependent effects. Theoretically, such distinctions should be discernible. In terms of clinical efficacy and safety, the ChE inhibitors are the best (Raschetti et al., 2007).

Rivastigmine, a reversible inhibitor of acetylcholinesterase and butyrylcholinesterase enzymes, is noted for its structure-specific action and limited peripheral side effects. It is used worldwide to treat various stages of Alzheimer's disease and was first approved to be marketed for AD (Mutlu and Degim, 2005). The interactions with other drugs of rivastigmine are minimal, which signifies its potential and makes it a good candidate for medication to be used in elderly individuals who have a coexisting disease or are on different medications (Raghavan et al., 2012). However, the limitation that intervenes with its oral use is its hydrophilic nature, which restricts its entry into the brain and entails its frequent dosing that can cause serious cholinergic side effects.

With the advent of nanocarriers, it became easy to deliver drugs directly to the targeted site and avoid their distribution to peripheral sites, leading to minimalistic side effects when compared to existing conventional dosage forms (Schwarz et al., 1994; Vashist et al., 2018). Several colloidal particulate delivery systems, such as magnetic nanoparticles, nanoemulsions or nanosuspensions, liposomes, and lipid particulate systems [e.g., solid lipid nanoparticles (SLNs) and nanostructured lipid carriers (NLCs)], have been investigated for delivery *via* N2B, with results indicating that they are effective because they are easily absorbed by nasal mucosa (Chouhan et al., 2015; Kaushik et al., 2018; Tiwari et al., 2019; Tomitaka et al., 2019; Nehra et al., 2021; Pawar et al., 2021). Providing larger drug loading and shielding from enzymatic metabolism results in enhanced selectivity, greater bioavailability, and longer pharmacological effect duration (Souto et al., 2004). SLNs have specific advantages over other nanoparticulate systems, including superior biocompatibility, ease of manufacture, and regulatory approval, all of which contribute to their biomedical utility (Kumar et al., 2008). These are lipid nanocarriers, which are spherical and their average diameter lies between 100 and 1,000 nm (Haque et al., 2012). Because of their lipophilic nature and other distinguishing qualities, such as sustained release, high drug loading capacity, good drug targeting efficiency (% DTE), and viability to surround or encapsulate multiple classes of drugs, SLNs have a significant advantage over other nanocarriers. It makes SLNs a viable conveyance vehicle for a wide range of pharmacological moieties that have difficulty traversing N2B (Lockman et al., 2004).

Pharmaceutical Quality by Design (QbD) is a systematic approach to development that starts with predefined goals and emphasizes product and process understanding and control based on sound science and risk management. This approach delivers product and process understanding for continuous improvement. Among its various diverse elements, the experimental designs are considered a pivotal tool, which provides maximal information using minimal experimentation. The use of the QbD technique has become a critical component of the pharmaceutical business. The goal of this technique is to determine the effect of critical process parameters (CPPs) and critical material attributes (CMAs) on critical quality characteristics. This approach states that quality is not inherited in the product, but is built in every step of the process. In this way, it ensures the predefined quality of the product during the designing, developing, and manufacturing of any product (Jain et al., 2008; Lionberger et al., 2008; Lawrence et al., 2014; Devi et al., 2022).

The originality of this work lies in the use of a combination of two modernized methods and easy-to-use equipment by optimizing and designing the experiment using the QbD approach (Xu et al., 2011). Also, the chosen combination of lipid and surfactant gave far better results with regard to entrapment efficiency, particle size, and drug release when compared to the previously reported methods of SLNs. The lower amounts of organic solvents utilized in the formulation process were removed using a Rota evaporator, demonstrating that the formulation is safe because no organic solvents are left behind, highlighting its superiority over other previously reported production processes (Lawrence, 2008; Bastogne, 2017).

In this study, RT-loaded SLNs for intranasal administration were developed using glyceryl monostearate, polysorbate 80 and 90% methanol by employing hot homogenization and a modified solvent-evaporation process. The formulation was optimized by the implementation of a central composite design. The optimized formulation was further evaluated for various parameters, such asparticle size, zeta potential, % entrapment efficiency, drug content, surface morphology, DSC, FTIR, *ex vivo* drug release, and stability studies. Thus, this study aimed to improve the pharmacokinetic profile and permeation rate of rivastigmine tartrate for the effective management of AD.

## Materials and methods

### Chemicals

Alembic Pharmaceuticals (Vadodra, Gujarat) sent a free sample of rivastigmine tartrate (RT). Sigma Aldrich, Bangalore, India, provided glyceryl monostearate (GMS) and polysorbate 80. Double distilled water (DDW), isopropyl alcohol (IPA), and analytical grade reagents were utilized.

### Instruments

*In vitro* profiling and thermal analysis of pure drug and produced SLNs were performed using a UV-Visible spectrophotometer (Shimadzu, UV-1800) and DSC Q200 (TA Instruments Trios V4.1, USA). The particle size (PS), zeta potential, and polydispersity index (PDI) were determined using Zetasizer (Malvern Zetasizer, Ver. 7.11). The transmission electron microscope (TEM) was used to study the morphology of the optimized formulation (H-7500, Hitachi Ltd., and Japan). A molecular weight cutoff of 12–14 kDa was used in *in vitro* research that involved the use of dialysis membranes (Himedia, Mumbai, India). Spectrum 400 FTIR/FIR Spectrometer, Perkin Elmer, and USA spectrophotometer were used in the FTIR (Fourier-transform infrared) investigation.

### Preliminary screening of lipid, solvent, and surfactant

#### Screening of lipid

Solubility studies of the drug in the lipid help in determining the encapsulating index of a drug in the lipid nanoparticles. There is a direct relationship existing between drug solubility and encapsulation efficiency (Makoni and Ranchhod, 2020; Verma and Kaushik, 2020).

The tendency of the lipid melts to solubilize the drug, which has a direct effect on the drug loading capacity (encapsulation efficiency) in the lipid, was the lipid selection criteria. Several lipids with better drug solubilizing potential were investigated, including GMS (Imwitor 900), stearic acid, cholesterol, and palmitic acid. RT (10 mg) was placed in a weighing vial for the lipid solubility tests (15 ml). The solid lipids were then individually heated to 5–10°C above their melting point. Gradually increasing volumes of melted lipid were added to the weighing container holding RT, which was then placed on the vortex mixer for continuous churning at a constant temperature. The amount of lipid melts necessary to solubilize RT (10 mg) was visually recorded. To avoid errors, the experiment was repeated three times, with the findings given as mean ± standard deviation (SD) (Peterson et al., 2009).

#### Screening of surfactant

In 1949, William C. (Bill) Griffin developed the hydrophilic–lipophilic balance (HLB) system. According to this system, lipids, surfactants, fats, or oils have a required HLB. The lipid selection was made based on the solubilizing potential of lipid for the drug (Azeem et al., 2009).

The selection of surfactant was done based on the HLB value of the selected lipid, i.e., GMS. GMS has the HLB value of 3.8, and therefore the HLB value of surfactant needed to emulsify the GMS for a stable emulsion should be around or more than 3.8. Hence, surfactant or co-surfactant or solvent should be chosen in such a concentration as to have a required combined value of 3.8 or more than 3.8 (Bhattacharya et al., 2022).

In this research work, several surfactants like polysorbate 80, Cremophor RH 40, and soya lecithin alone or in combination were used for the fabrication of SLNs. The stability of prepared SLN dispersion was observed visually after 24 h.

#### Screening of solvent

A random trial was done for screening different solvents to determine their solubilizing capacity for the chosen lipid. For this, an already known quantity of lipid was gradually added to 2 ml of each solvent with continuous stirring. The prepared samples were sealed and stirred for a fixed time. The endpoint of the experiment was observed visually when the solution appeared transparent. It signifies the capacity of the solvent to dissolve the lipid. Higher the capacity to solubilize, the better the solvent (Duong et al., 2020).

### Preparation and optimization of SLNs by central composite design

#### Preparation of RT-loaded SLN (RT-SLN)

The RT-SLNs are fabricated by an amalgamation of various techniques, including hot homogenization, modified solvent-evaporation diffusion method, and ultra-probe sonication technique (Lawrence, 2008). Various batches of formulations were made that were suggested by Design Expert^®^ software as demonstrated in Table 1. In brief, GMS was used as the solid lipid, and polysorbate 80 (hydrophilic surfactant) was adopted to reduce the interfacial tension between the lipid and drug. Initially, an aqueous surfactant solution heated to 3–5°C above the melting point of lipid was prepared. The chosen solid lipid (GMS) was melted at 60–65°C, to which drug (10 mg) and 5 ml of 90% of methanol solution were added under continuous stirring. In the aqueous surfactant solution prepared with the same temperature, a lipophilic phase containing drug was added to it. The nanoemulsion to be formed was stirred continuously at a temperature close to the melting point of the lipid used for 30 min at 10,000 rpm, and the organic solvent (methanol) used was removed by using a Rota evaporator (Joshi et al., 2010).

**Table 1:** Experimental runs designed by CCD and the obtained responses.

**F. Code**	**X1 (%)**	**X2 (%)**	**Y1 (nm)**	**Y2 (%)**	**Y3 (%)**
F1	2.00	2.00	110.50	81.25 ± 1.23	94.86 ± 1.12
F2	2.00	3.41	119.80	76.45 ± 0.14	89.67 ± 1.09
F3	3.41	2.00	140.30	85.62 ± 0.45	96.66 ± 0.56
F4	3.00	1.00	160.60	80.25 ± 0.66	93.22 ± 0.87
F5	0.59	2.00	80.80	60.12 ± 0.99	68.45 ± 1.65
F6	2.00	0.59	130.60	71.62 ± 0.77	71.25 ± 0.45
F7	1.00	1.00	87.80	64.25 ± 0.89	69.62 ± 0.99
F8	3.00	3.00	130.90	78.67 ± 0.99	91.68 ± 0.79
F9	2.00	2.00	112.50	80.35 ± 0.45	92.6 ± 0.34
F10	1.00	3.00	60.60	50.17 ± 0.34	40.66 ± 67
F11	2.00	2.00	123.30	85.28 ± 0.99	95.32 ± 0.79
F12	2.00	2.00	120.50	82.25 ± 0.68	95.43 ± 0.74
F13	2.00	2.00	130.10	83.68 ± 1.25	95.55 ± 0.54

The nanoemulsion obtained was sonicated afterward with a probe sonicator for 5 min at an amplitude of 60%. The nanoemulsion formed was then lyophilized to get the final nanopowder using mannitol as a cryoprotectant. The powder obtained was re-dispersed in a sufficient amount of water to obtain final dispersion, that is, RT-SLNs (Cavalu et al., 2020).

#### Optimization and statistical analysis of SLNs by central composite design

A central composite design (CCD) was used to choose the best experimental conditions using independent or autonomous variables with their coded levels and generating graphs of response surface by using statistical or mathematical models. The design process used was personalized by having a check on pre-decided independent factors and dependent variables with varied coded levels (Raza et al., 2013). They should be carefully screened and optimized to get an obligatory product. It gives the least required number of experiments to get appropriate results by optimizing the critical factors and estimating the interactions and quadratic effects of the dependent factors on the properties of RT-SLNs (Kutbi et al., 2021).

Lipid concentration (X1) and surfactant concentration (X2) were chosen as crucial factors based on the pre-optimization, and their effect on the dependent variables [particle size (Y1), entrapment efficiency (Y2), and drug release (Y3)] was assessed for the desired responses (Miere et al., 2022). Based on an extensive literature search, 13 runs, two coded factors, and three levels of CCD were used to optimize the formulation by altering the proportion of lipid (1–3%) and (Tween 80) surfactant (1–3%).

Herein, various statistical tests and methods have been used, which include variations in surfactant concentration and lipid concentration (Lionberger et al., 2008). These are the critical factors that influence particle size, % entrapment efficiency, and % drug release (Jain et al., 2008). In this research, the QbD approach has been put in an application for the optimization of solid lipid nanoparticle formulations that help in reducing the experimental runs by using the design of the experiment and generating a reliable set of conditions to work out the best formulation by using statistical and mathematical models. The statistical analysis of variables was done using the analysis of variance (ANOVA). The DoE software was utilized to select the best fit model based on sequential *p*-value, predicted R^2^, and adjusted R^2^ and lack of fit *p*-value (Aboti et al., 2014). Each factor showed their significant contribution based on F-value > 0.05 and *P*-value < 0.05 (Marto et al., 2016). The relationship between factors and responses is described by actual vs. predicted values, 2-D contour plots, and 3-D response surface plots. The polynomial equation with a positive and a negative sign of the coefficient's magnitude indicates the increasing and decreasing effect on the response, respectively (Dudhipala and Janga, 2017). To construct the polynomial equations and develop the models after reviewing their statistical significance, Design Expert^®^ software was used (Behbahani et al., 2017). The 2° polynomial equation constructed by the software for the response is given in **Eqn. 1**.


(1) $$\text{Y}=\text{B}0+\text{B}1\text{X}1+\text{B}2\text{X}2+\text{B}3\text{X}1\text{X}2+\text{B}4\text{X}1^{2}+\text{B}5\text{X}2^{2}$$

#### Selection of optimized formulation

Various parameters like high % encapsulation efficiency and optimum particle size with efficient % drug release were considered to get optimized RT-SLN. The optimization was done by studying the desirability plots based on the desirability function ranging from 0 to 1 with the use of a numerical technique. 2-D and 3-D response surface plots were obtained using the graphical method (Beg et al., 2019).

### Characterization of optimized formulation

#### Particle size and zeta potential determination

Zetasizer Ver. 7.11 (Malvern Instruments, UK) was used to determine the mean particle size, particle dispersion index (PDI), and zeta potential of the prepared SLN. The photon correlation spectroscopy technique measures the particle size of dispersing colloidal samples. It detects the average particle diameter and agglomeration or aggregation of particles that ultimately help in verifying the stability of prepared formulations (Verma et al., 2021). Using cells of 10 mm diameter set at an angle of 90°C at 25°C, the mean diameter of the created SLNs was determined. By dispersing the particles through electrostatic repulsion, the zeta potential evaluates the electrophoretic mobility of any colloidal system (Priyanka et al., 2018). All measurements were carried out by first diluting them with distilled water and removing the air bubbles by sonication. The readings were taken three times, and data were presented as mean ± S.D.

#### Percentage entrapment efficiency

The %EE of RT-loaded SLNs was determined by the cooling centrifuge method. The nanoparticles were placed in the refrigerated centrifuge at a high speed (C-24BL, Remi) at 10,000 rpm (4°C) for 30 min, and the supernatant was separated from the settled pellet of solid lipid nanoparticles (Rahman et al., 2019). The collected supernatant was examined after suitable dilution for free drug content at 263 nm by UV-Vis spectrophotometer. The % entrapment efficiency was calculated according to **Eqn. 2**.


(2) $$\%\;\text{EE}=\frac{\text{Total drug added}-\text{Unentrapped drug}}{\text{Total drug added}}$$

#### Drug content

To assess the drug content, approximately 0.1 ml of the produced RT-SLN was diluted in approximately 10 ml of methanol. The prepared mixture was sonicated and filtered through a 0.45 μm syringe filter (Vijaykumar et al., 2014). The solution was spectrophotometrically examined at 263 nm, and the drug content was estimated according to **Eqn. 3**.


(3) $$\text{Drug content}\;=\frac{\text{Amount of drug obtained}\;}{\text{Total drug added}}\text{X}\;100$$

#### Transmission electron microscopy

The surface morphological studies of RT-SLN were conducted using TEM (TEM, Hitachi H-7500, and Japan). The sample was diluted 20 folds (1/20) with pure water and placed onto a copper grid of 400 # that was previously coated with the copper film (Padhye and Nagarsenker, 2013). The analysis was performed by negatively staining the sample prepared with 1% phosphotungstic acid in the phosphate buffer of pH 7.4. Microscopy was carried out at an accelerated voltage of about 80 kV. The inspection of the sample was carried out after air drying (Pucek-Kaczmarek, 2021).

#### Differential scanning calorimetry

To investigate the enthalpy, physical, and chemical properties of RT, lipid, physical mixture, and RT-SLN, thermal analysis was performed. In RT-SLN, the DSC Q200 (TA Instruments Trios V4.1, USA) was employed to screen for potential drug–excipient (lipid) interactions. The samples were sealed in an aluminum pan and heated at a rate of 10°C per minute over a temperature range of 50–150°C. The analysis was carried out in two conventional aluminum pans, with 5 mg of sample in one pan and a reference pan in the other. The procedure was carried out under nitrogen purge at a flow rate of 50 ml/min (Singh et al., 2012; Verma and Kaushik, 2019).

#### Fourier-transform infrared spectroscopy

Infrared spectra of rivastigmine tartrate alone and when combined with excipients (i.e., lipid, surfactant, physical mixture, and formulation) were determined with FTIR-8400S instrument (Shimadzu Corporation) using previously reported KBr disk/pellet dispersion method (Cavalli et al., 1995). The samples for the testing process were made into compressed pellets by first grinding them with KBr powder (Seyed et al., 2017). The FTIR spectra were scanned across a range of 4,000–400 cm^−1^ (resolution 4 cm^−1^ /50 scans). The peaks were examined for any significant differences in the spectrum obtained for the plain drug, which included RT, GMS, Polysorbate 80, RT, and GMS, and a physical mixing of RT and GMS.

#### *In vitro* release study of RT-solid lipid nanoparticles

A comparative *in vitro* release study of RT-SLN and RT-Solution (RT-Sol) (10 mg of RT in aqueous surfactant solution alone) was performed by using Franz diffusion cell (Hanson Research–Telemodul 40 S, Chatsworth, CA) having a donor compartment and a receptor compartment of volume 20 ml. For the diffusion study, cellulose acetate membranes soaked in PBS 6.4 overnight were sandwiched between the two compartments and fixed using a tight clamp to prevent the leakage of media by diffusion (Zhang et al., 2010). Throughout the studies, the temperature of the cell was maintained at 37 ± 0.5°C, with a magnetic bead kept in the receptor compartment (PBS 6.4) for continuous stirring.

In comparative diffusion research, RT SLN dispersion (equal to 10 mg of drug) was initially placed in the donor compartment, followed by RT-Sol in triplicates. To maintain the sink conditions, aliquots of 1 ml were withdrawn at varied time intervals (0.5, 1, 2, 4, 6, 8, 10, and 24 h) using syringe tubing with the equal volume being replaced by PBS solution for each sample collected. The comparative release data obtained by the kinetic analysis were fitted to multiple kinetic models, including zero order, first order, Higuchi's equation, and Korsmeyer's–Peppas model.

#### *Ex vivo* diffusion of RT-SLN

An *ex vivo* diffusion study of RT-SLN solution was carried out in Franz diffusion cell to determine the permeation efficacy through the nasal mucosa. The diffusion cell having a donor compartment and a receptor compartment of volume of 20 ml was used. Fresh tissues from the nasal mucosa of the goat's nasal cavity were removed carefully, rinsed, and equilibrated with PBS (pH 6.4) for 20–30 min thoroughly. The excised nasal mucosa (thickness of 0.2 mm) was jammed between the receptor and donor compartments (mucosal side facing receptor compartment) after cutting to an appropriate size. The diffusion cell was thermostated at 37 ± 0.5°C. The temperature of the cell was thermostated at 37 ± 0.5°C throughout the studies with a magnetic bead kept in the receptor compartment (PBS 6.4) for continuous stirring (Yasir et al., 2014).

For comparative diffusion studies, RT-SLN dispersion (equivalent to 10 mg of drug) was initially placed in the donor compartment, followed by RT-Sol in triplicates. To maintain the sink conditions, aliquots of 1 ml were withdrawn at varied time intervals (0.5, 1, 2, 4, 6, 8, 10, and 24 h) using syringe tubing with equal volume replacement of PBS solution for each sample collected. At 263 nm, the diluted samples were spectrophotometrically evaluated for RT content. The amount of drug penetrated per unit area (g/cm^2^) vs. time (h) was plotted, and the slope yielded flux (g/cm^2^/h) and diffusion coefficients (cm^2^/h). The mean data for % medication diffused per unit skin surface area (g/cm^2^) vs. time were plotted after three measurements (h). The total amount of medication that penetrated *via* nasal mucosa was calculated according to **Eqn. 4**.


(4) $$\begin{array}{c} \text{Jss}/\text{C}0=\text{Kp} \end{array}$$

Equation 4 was used to compute the permeability coefficients (Kp, cm/min), where Jss is the steady-state flux and C0 is the initial drug concentration in the donor compartment.

#### Nasal histopathological studies

For performing a nasal histopathology study, fresh tissues from the nasal mucosa of a goat's nasal cavity were removed carefully, rinsed, and equilibrated with PBS (pH 6.4) for 20–30 min thoroughly. Nasal mucosa was cut into three pieces, and pieces with an even thickness (0.2 mm) were selected for the study. For 1 h, the three selected pieces were treated with negative control (PBS, pH 6.4), positive control (IPA), and RT-SLN. The dipped mucosa was dissected and stained using dyes (hematoxylin and eosin) after being given a proper wash with distilled water. The mucosa was dissected and examined with the help of an optical microscope (Magnus, India) at a magnification of 100X for the mucocilia by a pathologist to identify any visual damage to the mucosa (Hogan et al., 2020).

### Pharmacokinetic parameters and brain-targeting study

#### Pharmacokinetic studies

The study was conducted after the approval from IAEC (1355/PO/Re/L/10/CPCSEA) of M.M college of Pharmacy under Form B with protocol no. MMCP-IAEC-19.

For performing pharmacokinetic studies, male albino Wistar rats of age 6–8 weeks weighing 150–200 g were divided into three different sets: the first set was given RT-Sol intravenously (positive control), the second set was given RT-Sol intranasally (positive control), and the third set was given RT-SLN intranasally.

#### Plasma drug concentration estimation

The first set of rats was given drug solution (0.178 mg/ml) through the tail vein, whereas the second and third sets of Wistar rats were given the same concentration of drug intranasally (RT-Sol and RT-SLN, respectively) in the nostrils using a micropipette. For intranasal administration of drugs, rats were held firmly from the back in a slanting position to avoid dripping of solution by prior anesthetizing them with diazepam (Sharma et al., 2015; Yasir et al., 2017).

The rats were killed humanely by administering an overdose of pentobarbital sodium at different time intervals (0.5, 1, 2, 6, 8, and 12h) (*n* = 3 each time point per group), and the collected blood was centrifuged at a high speed (4,000 rpm/ 20 min) and supernatants from different aliquots were separated and stored at −21°C for drug content analysis using high-performance liquid chromatography (HPLC) (Narayan and Choudhary, 2017).

#### Brain drug concentration estimation

For simultaneous estimation of RT concentration in the brain, the rats were killed humanely at the same time intervals to separate the brain, and the brain was rinsed two times with normal saline. To it, cold saline solution was added and homogenized on ice, and the collected blood sample was centrifuged at a high speed (4,000 rpm/20 min) and supernatants from different aliquots were separated and stored at −21°C for the analysis of drug content using HPLC (Van Holde et al., 2006). Statistical analysis was done using Kinetica^®^ software (Thermo scientific). All results were expressed as mean±standard deviation. The difference among the groups was compared with ANOVA. *P*-value < 0.05 was considered statistically significant.

### Stability studies

To study the stability profile of the drug and to check the physicochemical stability of the prepared formulation, it was kept under specified storage conditions of temperature and relative humidity. The stability study of the optimized SLN was performed in triplicate. Optimized SLNs were kept at 4 ± 2°C (refrigerator), 25 ± 2°C/60 ± 5% RH, and 40 ± 2°C/ 75 ± 5% in a stability chamber (Hicon instruments, New Delhi). The samples were analyzed for various parameters like PS, zeta potential, PDI, %EE, and DR% at an interval of initial, 1, 3, and 6 months.

## Results and discussion

### Preliminary screening

#### Selection of lipid

Results of the solubility experiment indicated that amongst the GMS, cholesterol, palmitic acid, and stearic acid, the GMS had a higher potential to solubilize the RT, as shown in Supplementary Figure S1. Also, the biocompatibility and acceptability of GMS from the nose to the brain have been proven as per previous literature. This entailed the selection of GMS in the present study.

#### Selection of surfactant

The selection of the surfactant was mainly determined by the HLB value of the lipid. SLN dispersion prepared in polysorbate 80 was stable when compared to other surfactants alone or in combination after 24 h. Hence, polysorbate 80 was selected as a surfactant in this study. Its applicability and safety profile have been proven in the previous literature, which further favored its selection (Singh et al., 2012).

#### Selection of solvent

Lipid solubility in different solvents was the main selection criteria for a solvent. Methanol showed the highest solubility of lipid when compared to chloroform, ethanol, and ethyl acetate. Also, it was found to be non-toxic when used in permissible quantities.

### Preparation and optimization of SLNs by central composite design

#### Preparation of SLNs

Various batches of formulations were made as suggested by Design Expert^®^ software. RT-loaded SLNs were prepared by a combination of modified solvent-evaporation diffusion method and probe sonication technique.

#### Optimization and statistical analysis of SLNs by central composite design

A 13-run face-centered central composite design was used to minimize the particle size, maximize the %EE and %DR. The independent variables, such as X1 and X2, have a significant effect on the dependent variables PS (Y1), %EE (Y2), and DR% (Y3), which were calculated by regression analysis. The regression analysis generated a linear model equation for PS and a quadratic 2° polynomial equation for %EE and %DR. The model suitability of PS was dependent on the significance of two variables that were selected during preliminary analysis, such as the amount of lipid (GMS) and amount of surfactant (polysorbate 80). The results obtained through ANOVA for selected responses (Y1, Y2, and Y3) are given in Table 2. Actual vs. predicted graphs, 2-D contour plots, and 3-D response surface graphs for selected responses Y1, Y2, and Y3 are given in Figures 1–3.

**Table 2:** ANOVA for response surface quadratic model for checking model suitability for Y1, Y2, and Y3.

**ANOVA**	**Sum of squares**	**DF**	**Mean square**	**F value**	***P*** **-value**	**Model**
Y1	7,106.20	2	3,553.10	26.49	0.0001	Significant
Y2	1,280.37	5	256.07	12.82	0.0021	Significant
Y3	2,733.84	5	546.77	5.67	0.0209	Significant

**Figure 1:** Actual vs. predicted values for **(A)** particle size, **(B)** % entrapment efficiency, and **(C)** *in vitro* drug release.

**Figure 2:** 2-D contour plots for **(A)** particle size, **(B)** % entrapment efficiency, and **(C)** *in vitro* drug release.

**Figure 3:** 3-D response surface graphs for **(A)** particle size, **(B)** % entrapment efficiency, and **(C)** *in vitro* drug release.

##### Statistical analysis of particle size (Y1)

It was observed that (*p* < 0.05) for the model was highly significant and could predict the closest response value of PS. The *p*-value for lack of fit was found to be greater than 0.05, which makes it marginally insignificant. The obtained value for “lack of fit” was 2.8, which states that there was only a 1.3% chance for it to be greater and it can result due to the appearance of noise. From the obtained equation, it was found that the positive coefficient (28.41) of X1 (amount of lipid) had a direct effect on particle size. Positive coefficient of X2 was showing that increasing surfactant concentration tends to increase particle size, negative coefficient of X2 (amount of surfactant) was showing that increasing surfactant concentration tends to reduce particle size as shown in **Eqn. 5**.


(5) $$\begin{array}{c} \text{Y}1(\text{PS})=116.02+28.41\text{X}1-9.02\text{X}2 \end{array}$$

Thus, we can assume that the amount of lipid (GMS) has a positive effect and the amount of surfactant (polysorbate 80) has a negative effect on the PS.

##### Statistical analysis of entrapment efficiency

It was observed that *p* < 0.05, which states that the model was highly significant and can predict the closest response value of %EE. The *p*-value for lack of fit was greater than 0.05, which makes it marginally insignificant. The obtained value for “lack of fit” was 10.82, which states that there was only a 2.1% chance for it to be greater only if noise occurs. Also, X1 is the amount of lipid with *p* < 0.0001, and X12 (2° effect of X1) with *p* < 0.05 had a significant value.


(6) $$\begin{array}{l} \begin{array}{ccc} \text{Y}2(\%\text{EE}) & = & 82.56+10.07\text{X}1+1.10\text{X}2-3.13\text{X}1.\text{X}2 \end{array}\\ \;-\;6.13\text{X}1^{2}-5.54\text{X}2^{2} \end{array}$$

While looking at the polynomial equation obtained as shown in **Eqn. 6**, it was observed that the positive coefficient (10.07) of X1 (amount of lipid) also has a direct relationship with %EE. %EE increases with increasing lipid concentration and surfactant concentration. The reason may be the extra space created by acylglycerols mixtures for the drugs to get enclosed, and the use of polysorbate 80 increased the film strength of the formulation (Zhang et al., 2010). In addition, the significance of the negative coefficient of X1X2 showed that increasing surfactant concentration may alter the function of lipid and polysorbate 80 and tend to decrease their effect on entrapment efficiency.

##### Statistical analysis of % drug release

It was observed that *p* < 0.05, which states that the model was highly significant and can predict the closest response value of %DR. The *P*-value for lack of fit was greater than 0.05, which makes it marginally insignificant. The obtained value for “lack of fit” was 14.24, which states that there was only a 2.5% chance for it to be greater in the case of the appearance of noise. Also, X1 with *p* < 0.0001 and X12 (2° effect of X1) with *p* < 0.05 had a significant value.


(7) $$\begin{array}{l} \begin{array}{ccc} \text{Y}3(\%\text{DR}) & = & 94.75+14.31\text{X}1+0.5563\text{X}2-6.86\text{X}1.\text{X}2 \end{array}\\ \;-\;8.03\text{X}1^{2}-9.07\text{X}2^{2} \end{array}$$

While looking at the polynomial equation obtained as shown in **Eqn. 7**, it was observed that the amount of lipid (X1) has a positive effect on DR%, and the amount of surfactant (X2) may have a slight positive effect on DR%. The reason could be the same as for entrapment efficiency, that is, increasing the surfactant concentration up to a certain limit will help in increasing the drug release, and after a certain point, drug release will decrease. This could be explained by the fact that surfactant has reached its critical micelle concentration and will lead to the formation of micelles. The interaction factor X1X2 of lipid and surfactant also justifies the point that when lipid and surfactant are used in an optimum amount, they will give a good drug release profile, while the second-order terms signify the negative effect of the overuse of independent factors.

Thus, the maximum DR% was found with an increased level of lipid and lower level of surfactant used, as can be seen from the graphs. Hence, it can be stated that both the factors affect the DR%, i.e., the amount of lipid (GMS) has a directly proportional effect and the amount of surfactant (polysorbate 80) has a slightly positive effect on the DR%.

#### Selection of optimized formulation

The optimization of the formulation was done by desirability index. Formulation 1 was found to be the optimum formulation considering all the dependent parameters as shown in Figure 4, which include lipid (2%) and surfactant (2%). The observed values for Y1, Y2, and Y3 of the optimized batch were found to be 110.2 nm, 81.25 ± 1.233%, and 94.86 ± 1.124%, respectively, which were very close to the predicted values. Furthermore, *in vitro* drug release studies, *ex vivo* permeation studies, DSC, FTIR, and morphological and stability studies were carried out for the optimized batch.

**Figure 4:** Desirability index for dependent variables.

### Characterization of optimized formulation

#### Particle size and zeta potential

The zeta potential of the solid lipid nanoparticles explains the storage stability conditions of the prepared formulation. Zeta capability indicates the degree of electrostatic repulsion between adjoining, similarly charged particles in dispersion (Cavalli et al., 1995). The particle size of the optimized SLN batch was 110.2 nm with a PDI value of 0.309, as shown in Figure 5. These results revealed uniform distribution of the nanosize particles of the developed formulation.

**Figure 5:** Particle size of optimized formulation.

The ZP value of the optimized formulation was found to be −28 ± 1.5 mV, as shown in Supplementary Figure S2. The addition of polysorbate 80, which is a non-ionic surfactant, stabilized the emulsion due to steric repulsion. The presence of a negative charge on the interface of SLNs will cause double-layer repulsion between the formed droplets and prevent their agglomeration by strong repulsive forces during storage.

#### Percentage EE

It is generally reported that increasing or decreasing the surfactant concentration affects the EE. When the polysorbate 80 concentration was raised from 1 to 2% along with the increase in the lipid concentration from 1 to 3%, there was a sluggish decrease in the particle size, but the EE improved appreciably. This may be due to the surfactant enclosing the lipid particle and escaping the drug leakage. The %EE of optimized SLN formulation was found to be 82.56 ± 0.42%.

#### Drug content

There was no degradation of the drug during the preparation of SLN, and the drug content of the optimized formulation was found to be 99 ± 0.56%.

#### Transmission electron microscopy

The TEM analysis of RT-SLN revealed the morphology of the prepared RT-SLN. SLNs were found to be spherical in shape, and the size distribution was found to be in the range of 50–150 nm as shown in Figure 6. This finding further confirmed the uniform size distribution as shown by Zetasizer.

**Figure 6:** TEM image of optimized RT-SLN formulation.

#### Differential scanning calorimetry

Differential scanning calorimetry is a thermoanalytical technique that is used to investigate the enthalpy change as a function of the temperature of crystalline material. DSC thermograms were recorded for pure drug (RT), lipid (GMS), lyophilized RT-SLN, and physical mixture (RT + GMS + polysorbate 80), as shown in Figure 7. The recorded thermogram of RT-SLN did not show the melting peak of SLN crystals. A sharp intact endothermic peak at 60.9°C was observed, which states that RT-SLN has transitioned from crystalline to an amorphous state, as shown in Figure 7C. These illustrations agree with the results obtained from the FTIR spectrum, which also proved the entrapment of RT in the matrix of GMS. The separate melting endothermic peaks of RT and GMS in their physical mixture (Figure 7D) confirmed their crystalline nature and compatibility with each other.

**Figure 7:** DSC thermogram of **(A)** RT, **(B)** GMS, **(C)** optimized RT- SLN, and **(D)** physical mixture.

#### Fourier-transform infrared spectroscopy

The FTIR spectra obtained for a pure drug (RT), surfactant (Tween 80), lipid (GMS), physical mixture (RT+GMS+Tween 80), and SLN formulation are shown in Figure 8.

**Figure 8:** FTIR spectra of **(A)** RT, **(B)** polysorbate 80, **(C)** GMS, **(D)** physical mixture, and **(E)** optimized RT-SLN formulation.

The RT-SLNs showed the characteristic peaks at 3,417.42 cm^−1^, 1,692.16 cm^−1^, 1,402.76 cm^−1^, 1,073.84 cm^−1^, 506.67 cm^−1^, and 449.32 cm^−1^. The presence of characteristic peaks both inside the physical combination (drug and lipid) and drug-loaded SLN revealed that there was no noticeable physicochemical interaction between the drug and the lipid in the system.

#### *In vitro* study

The comparative *in vitro* release study of RT-Sol and optimized formulation (F1) was performed. The release of RT from the RT-Sol was nearly 95% within 6 h, whereas SLN formulation (F1) maintained the sustained release of the drug up to 94.86 ± 1.124% for 24 h. Initially, the percentage of drug diffusion in the case of RT-Sol was found to be higher when compared to the optimized formulation. The presence of the adsorbed drug on the surface of nanoparticles caused an initial quick release of the drug in the case of RT-SLN, which was followed by continuous release.

The release of integrated drugs from the interior of the homogeneous matrix of the nanoparticles was demonstrated by the continuous release of the drug. It also gives an idea about diffusion rate of drug from SLNs surrounding solid lipid shell's limiting effects. DSC data also highlights the low enthalpy requirement for RT entrapped within the lipid matrix (RT-SLN) than lipid only (GMS). It confirms the imperfect crystal lattice of the lipid, which leads to higher diffusion in the case of SLN through which the drug is diffused out (Joshi et al., 2010). The value of R^2^ kinetics confirmed that the release kinetics of RT-SLN (F-1) follow the Higuchi model rather than the zero-order or first-order kinetics as depicted in Supplementary Figure S3.

#### *Ex vivo* study

*Ex vivo* diffusion study of RT-Sol and RT-SLN (F1) was performed using nasal mucosa of goat (biological membrane) that simulated *in vivo* barrier. Cellulose acetate membranes used in *in vitro* studies are artificial membranes, so we cannot rely on the findings obtained from *in vitro* studies. Figure 9 shows the flux and diffusion coefficients for RT-SLN and RT-Sol as 3.378g cm^−2^ h^−1^ and 0.310 cm^−2^ h^−1^, respectively. A higher value of flux and diffusion coefficient in the case of RT-SLN highlights the higher penetration potential of lipidic nanoparticles, which further increased the solubilization tendency of the drug in the lipoidal membrane when compared to RT-Sol (Joshi et al., 2010). Also, the presence of surfactants worked as penetration enhancers and increased the permeability through the nasal mucosa, whereas RT-Sol has a low tendency to cross the lipoidal membrane owing to its hydrophilic nature.

**Figure 9:** *Ex vivo* study of optimized formulation.

#### Nasal histopathology study

A nasal histopathology study was performed on the nasal mucosa of a goat to study the nasociliary damage caused by various excipients used in the formulation of RT-SLN. The first piece of the nasal mucosa was treated with negative control (PBS, pH 6.4) that showed no nasociliary damage, while the second piece that was treated with positive control (IPA) showed damaged cilia lining which was indicated through the shedding of epithelial cells of the nasal membrane, as shown in Figure 10. Unlike positive control, the third piece treated with RT-SLN showed no visible signs of damage to the cilia of the nasal membrane, indicating the safety of the nasal administration of RT-SLN in humans. In addition, the pH of RT SLN was 5.8, which was within the range of human nasal pH (5–6.5).

**Figure 10:** Nasal histopathology studies of nasal mucosa **(A)** treated with PBS, **(B)** treated with IPA, and **(C)** treated with RT SLN. Magnification power (10x * 10x = 100X).

### Analysis of pharmacokinetic studies

After the administration of (a) RT sol (i.v.), (b) RT sol (i.n.), and (c) RT-SLN (i.n.), PK investigations were undertaken, and blood samples were evaluated for drug concentration using the RP-HPLC method in blood and brain. Figure 11 depicts the compartmental distribution of the drugs. In Tables 3, 4, the results of several PK parameters and compartmental distribution of drugs are presented, respectively. The *p*-values for C_max_, T_max_, and AUC_0−24_ were found to be <0.0001, which were extremely significant.

**Figure 11:** Illustration of compartmental distribution of RT-SLN (i.n.) and RT solution after i.n. and i.v. administration.

**Table 3:** Results of various pharmacokinetics parameters of RT-SLN (i.n.) and RT solution after i.n. and i.v. administration (*n* = 3).

**PK** **parameters**	**Type of formulation/route of administration**					
	**RT-Solution** ***i.v***.		**RT-Solution** ***i.n***.		**RT-SLNs** ***i.n***.	
	**Brain**	**Plasma**	**Brain**	**Plasma**	**Brain**	**Plasma**
*C*_max_ (ng/ml)	49.64 ± 5.58	78.5 ± 3.46	65.24 ± 3.35	71.79 ± 2.98	73.99 ± 5.66	62.49 ± 6.23
*T*_max_ (h)	1.00	0.50	1.00	0.67	0.67	2.00
AUC_(0−24)h(ng·*h*/*ml*)_	6,856.25 ± 14.46	9,066.21 ± 13.78	9,876.34 ± 11.62	12,016.6 ± 12.90	20,256.49 ± 36.60	12,047.55 ± 34.78
AUC_(0−∞)__(*ng*·*h*/*ml*)_	7,018.40 ± 20.97	9,724.78 ± 45.67	12,567.76 ± 13.80	13,985 ± 34.85	25,678 ± 56.67	25,696.11 ± 23.90
AUMC_(0−24)h(ng·*h*2/*ml*)_	6,5895.50 ± 23.78	73,683.98 ± 32.67	78,967.67 ± 16.61	80,887.5 ± 21.90	184,334.059 ± 31.7	72,895.56 ± 12.90
AUMC_(0−∞)__(*ng*·*h*2/*ml*)_	8,7467.32 ± 23.67	90,756.724 ± 12.87	19,678.56 ± 45.78	20,018.998	11,789.89 ± 23.89	12,050.19 ± 12.90
*K*e _(h_^−1^)	0.10404	0.123041	0.12506	0.14855	0.09009	0.165

**Table 4:** Compartmental distribution of RT-SLN (i.n.) and RT solution after i.n. and i.v. administration (*n* = 3 ± S.D).

**Formulation**	**Sample**	**0.1 hr (ng/ml)**	**0.5 hr (ng/ml)**	**1 hr (ng/ml)**	**2 hr (ng/ml)**	**4 hr (ng/ml)**	**8 hr (ng/ml)**
RT-Sol i.v.	Brain	34.56 ± 4.78	42.78 ± 3.98	49.64 ± 5.58	40.89 ± 7.98	29.66 ± 6.98	19.15 ± 3.89
	Blood	70.89 ± 4.99	78.54 ± 3.46	76 ± 6.66	50.55 ± 7.67	40.90 ± 2.90	40.80 ± 1.70
RT-Sol i.n	Brain	37.99 ± 6.98	50.78 ± 7.98	65.24 ± 3.35	55.65 ± 6.12	50.43 ± 1.35	35.43 ± 5.90
	Plasma	47.32 ± 5.67	70.59 ± 2.98	63.08 ± 1.78	50.98 ± 3.09	45.67 ± 4.89	33.91 ± 3.88
RT-SLN i.n	Brain	62.26 ± 4.65	73.99 ± 5.66	65.11 ± 5.1	63.43 ± 1.98	55.37 ± 3.23	42.90 ± 1.78
	Plasma	50.13 ± 2.78	55.36 ± 2.61	58.44 ± 6.51	62.49 ± 6.23	49.89 ± 8.45	38.99 ± 2.64
RT-Sol i.v.	Brain/Blood	0.49	0.54	0.65	0.81	0.73	0.72
RT-Sol i.n	Brain/Blood	0.81	0.72	1.03	1.09	1.10	1.04
RT-SLN i.n	Brain/Blood	1.24	1.34	1.11	1.09	1.11	1.10

Various PK parameters that were evaluated in this study were as follows: C_max_ (ng/ml), T_max_ (h), AUC _(0−24)h_, AUC _(0−)h_, AUMC _(0−24)h_, AUMC _(0−)_, Ke _(h−1)_, and MRT (h). The statistical analysis was done using ANOVA. When compared to RT-Sol (i.n.) and RT-Sol (i.v.), RT concentrations in the brain after the intranasal administration of RT-SLN were shown to be relatively high at all periods of time (*p* = 0.05), as shown in Figure 11. In comparison to the brain, the concentration of RT in the plasma after intranasal delivery of SLN was low. The medication may be present in the plasma because of the i.n. route, which can lead to systemic absorption. Because of the direct nose-to-brain transfer following intranasal injection, the T_max_ for the brain is 0.667 h, while it is 2 h for plasma. When RT-SLN was delivered intranasally, the C_max_ value for the brain was 73.995.66 ng/ml, which was significantly higher than when RT-Sol was supplied intranasally and intravenously. It could be attributed due to the direct transport of the drug after crossing the blood–brain barrier. A similar result was reported by Barakat et al. (2005), who studied the absorption of carbamazepine after intranasal administration.

The value of AUC _(0−∞)*h*_ was found to be higher for RT-SLN administered intranasally when compared to RT-Sol given through i.v. and i.n. routes. The value of Ke for RT-SLN in the brain was found to be lower when compared to drug solutions given through other routes, highlighting its greater MRT, long half-life, and ultimately lower clearance and Vss. Also, the value of AUC_(0−∞)_ for RT-SLN in the brain was found to be twice that of RT-Sol given intranasally and thrice for RT-Sol given intravenously. The brain/blood ratios for RT-SLN were found to be high at all time points than RT-Sol given through i.n. and i.v. routes, signifying a higher drug targeting potential of SLN. Similar findings were reported by Qizhi et al. (2004) and Fazil et al. (2012). The study revealed that the drug uptake into the brain from the nasal mucosa mainly occurs *via* two different pathways. One is the systemic pathway where some amount of the drug is absorbed into the systemic circulation and subsequently reaches the brain by crossing the BBB. An optimized rivastigmine tartrate SLN-loaded transdermal film was successfully developed by Ravi and co-workers, which could control the release and permeation of rivastigmine tartrate up to 24 h (Ravi and Gupta, 2017). The lipophilic character of SLN helped in greater penetration of RT into the brain.

### Stability studies

Stability studies were conducted for 6 months to check the particle size, zeta potential, PDI, %EE, and %DR at 4 ± 2°C, 25 ± 2°C /60 ± 5% RH and 40 ± 2°C /75 ± 5% RH. It was observed that there was no significant change when the SLNs were kept at 4 ± 2°C and 25 ± 2°C/60 ± 5% RH, but the particle size increased significantly due to the aggregation at 40 ± 2°C/75 ± 5% RH, as shown in Table 5.

**Table 5:** Results of stability studies of optimized RT-SLN formulations (*n* = 3).

**Temp** **(°C)/RH (%)**	**Time** **(Months)**	**Characteristics parameter**				
		**Particle** **size (nm)**	**PDI**	**Zeta potential (mV)**	**% Entrapment** **efficiency**	**% Drug** **release**
4 ± 2	0	112.34 ± 3.96	0.303	−28.6 ± 1.7	82.53 ± 2.94	96.61 ± 0.85
	1	118.34 ± 2.87	0.316	−25.5 ± 1.2	81.3 ± 2.72	95.41 ± 0.56
	3	124 ± 3.56	0.378	−26.6 ± 1.9	80.33 ± 1.84	95.12 ± 0.32
	6	137 ± 1.59	0.463	−25.6 ± 1.4	80.53 ± 1.93	94.61 ± 1.41
25 ± 2/ 60 ± 5	0	112.34 ± 3.96	0.303	−28.6 ± 1.7	82.53 ± 2.94	96.61 ± 0.85
	1	118.34 ± 2.87	0.316	−25.5 ± 1.2	81.3 ± 2.72	95.41 ± 0.56
	3	124 ± 3.56	0.342	−26.6 ± 1.9	80.33 ± 1.84	95.11 ± 0.32
	6	140 ± 1.59	0.463	−25.6 ± 1.4	80.73 ± 2.30	94.61 ± 0.41
40 ± 2/ 75 ± 5	0	112.34 ± 3.96	0.383	−28.6 ± 1.7	82.53 ± 2.70	96.61 ± 0.85
	1	120.34 ± 2.17	0.416	−25.5 ± 1.2	81.3 ± 2.72	94.41 ± 0.19
	3	269.12 ± 3.26	0.578	−19.6 ± 1.9	80.33 ± 1.64	92.11 ± 0.13
	6	340.45 ± 1.59	0.663	−0.9 ± 1.4	81.30 ± 1.12	93.61 ± 0.49

The results indicated that there was negligible change in zeta potential, highlighting the physical stability of the formulation when kept at 4 ± 2°C and 25 ± 2°C/60 ± 5% RH, but a significant drop in the values was found after 3 months when kept at 40 ± 2°C/75 ± 5% RH, probably due to the removal of the outer coating of SLN as a result of aggregation of SLNs at a high temperature and humidity. There were non-significant changes in %EE and DR%. PDI was stable throughout the period at room temperature conditions and refrigerated conditions. However, it increased significantly under accelerated conditions, and the heterogeneity may be probably due to increased temperature conditions.

## Conclusion

Preformulation, lipid solubility, and drug excipient compatibility studies helped in the selection of a suitable lipid and surfactant, while trial batches helped in selecting their effective concentrations (refer Figure 12 for the summary). The central composite design was employed for choosing an optimized formulation and studying the effect of independent variables on the dependent ones. The particle size, %EE, and %DR of optimized formulation were reported as 110.2 nm, 82.56 and 94.86%, respectively. Morphology of the prepared SLN revealed the spherical shape, while the *in vitro* and *ex vivo* studies confirmed the controlled and sustained drug release from the optimized formulation. Nasal histopathology investigations confirmed that the optimized formulation was safe to consume intranasally, while the pharmacokinetic studies demonstrated the justification for enhanced bioavailability of the optimized formulation that is given intranasally. Stability studies demonstrated that the developed SLN was stable when stored under various storage conditions according to ICH recommendations. Hence, the SLN approach could be an appropriate and potential carrier for the transport of drugs to the target brain.

**Figure 12:** Schematic representation of development and evaluation of SLNs for intranasal route.

## Data availability statement

The original contributions presented in the study are included in the article/Supplementary material, further inquiries can be directed to the corresponding author/s.

## Ethics statement

The animal study was reviewed and approved by IAEC (1355/PO/Re/L/10/CPCSEA) of M.M college of Pharmacy under Form B with protocol no. MMCP-IAEC-19.

## Author contributions

DA, SB, and MK: conceptualization. DA: methodology. RV: software. DK: validation. SB: formal analysis. RV, SSA, DK, NK, GB, and SA: data curation. DA and RV: original draft preparation. AT, VM, VT, YT, RKS, and AA: reviewing and editing. SB and MK: supervision. All authors contributed to editorial changes in the manuscript and read and approved the final manuscript.

## Conflict of interest

Author RS is honorary-based associated with the iGlobal Research and Publishing Foundation (iGRPF), India. YT was employed by Zeon Lifesciences Pvt. Ltd. Author AA holds an unpaid position on the scientific board of the company AFNP Med Austria. The remaining authors declare that the research was conducted in the absence of any commercial or financial relationships that could be construed as a potential conflict of interest.

## Publisher's note

All claims expressed in this article are solely those of the authors and do not necessarily represent those of their affiliated organizations, or those of the publisher, the editors and the reviewers. Any product that may be evaluated in this article, or claim that may be made by its manufacturer, is not guaranteed or endorsed by the publisher.

## Supplementary material

Supplementary Figure S1 Solubility of drug in various lipids.

Supplementary Figure S2 Zeta potential of optimized formulation.

Supplementary Figure S3 Drug release kinetics of optimized RT-SLN.

## Abbreviations

ANOVA: Analysis of variance
CCD: Central composite design
DSC: Differential scanning calorimetry
FTIR: Fourier transform infrared spectroscopy.
